The article "Haematococcus pluvialis Carotenoids Enrich Fractions Ameliorate Liver Fibrosis Induced by Thioacetamide in Rats: Modulation of Metalloproteinase and Its Inhibitor" was published in 2021. Journal: Biomed Res Int.

# *Haematococcus pluvialis* Carotenoids Enrich Fractions Ameliorate Liver Fibrosis Induced by Thioacetamide in Rats: Modulation of Metalloproteinase and Its Inhibitor

**DOI:** 10.1155/2021/6631415

**Published:** 2021-02-11

**Authors:** Farouk K. El-Baz, Abeer Salama, Sami I. Ali, Rania Elgohary

**Affiliations:** ^1^Plant Biochemistry Department, National Research Centre (NRC), 33 El Buhouth St. (Former El-Tahrir St.), 12622 Dokki, Cairo, Egypt; ^2^Pharmacology Department, National Research Centre (NRC), 33 El Buhouth St. (Former El-Tahrir St.), 12622 Dokki, Cairo, Egypt; ^3^Narcotics, Ergogenics and Poisons Department, National Research Centre (NRC), 33 El Buhouth St. (Former El-Tahrir St.), 12622 Dokki, Cairo, Egypt

## Abstract

Hepatic fibrosis is a consequence of chronic liver diseases. Metalloproteinase and its inhibitor have crucial roles in the resolution of liver fibrosis. The current relevant study is aimed to evaluate the therapeutic effect of *Haematococcus pluvialis* (*H. pluvialis)* extract, astaxanthin-rich fraction, astaxanthin ester-rich fraction, and *β*-carotene-rich fraction as well as their mechanisms of action in curing hepatic fibrosis induced by thioacetamide (TAA). Liver fibrosis was induced using TAA (intraperitoneal injection, two times a week for 6 weeks), in a rat model and *H. pluvialis* extract (200 mg/kg), and other fractions (30 mg/kg) were orally administered daily for 4 weeks after the last TAA injection. Based on HPLC analysis, *H. pluvialis* extract contains *β*-carotene (12.95 mg/g, extract) and free astaxanthin (10.85 mg/g, extract), while HPLC/ESI-MS analysis revealed that *H. pluvialis* extract contains 28 carotenoid compounds including three isomers of free astaxanthin, *α* or *β*-carotene, lutein, 14 astaxanthin mono-esters, 5 astaxanthin di-esters, and other carotenoids. *H. pluvialis* and its fractions reduced liver enzymes, nitric oxide, collagen 1, alpha-smooth muscle actin, and transforming growth factor-beta as well as elevated catalase antioxidant activity compared to the TAA group. Also, *H. pluvialis* extract and its fractions exceedingly controlled the balance between metalloproteinase and its inhibitor, activated Kupffer cells proliferation, and suppressed liver apoptosis, necrobiosis, and fibrosis. These findings conclude that *H. pluvialis* extract and its fractions have an antifibrotic effect against TAA-induced liver fibrosis by regulating the oxidative stress and proinflammatory mediators, suppressing multiple profibrogenic factors, and modulating the metalloproteinase and its inhibitor pathway, recommending *H. pluvialis* extract and its fractions for the development of new effective medicine for treating hepatic fibrosis disorders.

## 1. Introduction

Liver fibrosis is induced by a chronic hepatic insult and associated with liver dysfunction and life-threatening complications [1]. Chronic liver diseases affected millions of patients worldwide; 30% of patients are likely to develop fibrosis and cirrhosis. Also, this condition is evolved towards liver cancer and an elevation in the mortality rate [2, 3]. In fibrosis and chronic liver diseases, there is an accumulation of fibrillar extracellular matrix (ECM) [4] and stimulation of sinusoidal endothelial cells releasing cytokines and activating hepatic stellate cells (HSCs) [5]. Also, Kupffer cells, hepatic macrophages, play an important role in the resolution of liver fibrosis [6] via the production of a large spectrum of matrix metalloproteinase (MMPs) expression [7]. MMP9 is a gelatinase enzyme produced by Kupffer cells and is implicated in the pathological process of hepatic injury [8]. The presence of MMP9 suppressed transforming growth factor-beta (TGF-*β*1) activation and reduced ECM components accumulation as collagen 1 and *α*-Smooth muscle actin (*α*-SMA) during fibrogenesis in the liver [9]. The expression MMP9 was elevated during fibrosis resolution in Kupffer cells [10]. In the liver fibrogenesis process, the most critical cytokine involved is TGF-*β* [11]. TGF-*β*1 can also control MMPs and tissue inhibitors of matrix metalloproteinase (TIMPs) expression. MMPs carry out an important function in degrading ECM components, and TIMPs have the ability to adverse MMP function [12, 13].

Carotenoids including *β*-carotene and astaxanthin showed abundant awareness lately due to their powerful antioxidant properties that trigger the protection of the organism against different oxidative stresses related disorders. Different carotenoids accumulate primarily in the liver, then they are transported by divers lipoproteins for releasing to the blood circulation from which it deposited in some organs and tissues including skin, kidneys, adrenal glands, adipose tissues, testes, and the prostate [14]. The accumulation of these carotenoids as antioxidants and their different metabolites in the liver can improve the hepatocyte metabolism and regulate the cellular oxidative conditions in certain liver complications [15] Astaxanthin is one of the most potent active carotenoids exhibiting an antioxidant effect 10 times greater than *β*-carotene and 100 times stronger than vitamin E, and it exists mostly in the form of fatty acid esters such as that produced by the microalgae *H. pluvialis*. Besides, astaxanthin and astaxanthin esters *H. pluvialis* microalgae synthesized *β*-carotene [16]. As a result of their potent competency to scavenge different reactive oxygen species and quench singlet oxygen, the antioxidant capability of different carotenoid individuals, including astaxanthin and *β*-carotene, is of prominent importance to human health [17] through their ameliorative ability against oxidative stress; the main promoter of many diseases including liver disorders [18, 19].

The health advantages of supplements containing *H. pluvialis* extract enrich in astaxanthin and astaxanthin esters have been the hot topic of several *in vitro* and clinical studies because of its potent antiaging influence, anti-inflammatory, gastroprotective, immunoprotective, cardioprotective, nephroprotective, neuroprotective, antiasthmatic, antidiabetic, and anticancer properties [20–23]. Besides astaxanthin, *β*-carotene has anticancer activity especially against lung and prostate cancers [24]. *β*-Carotene also has anti-inflammatory potentials by suppressing different proinflammatory markers including redox-based nuclear factor-kappa-*β* (NF-*κβ*), NADPH oxidase protein, inducible nitric oxide synthase (iNOS), and cyclooxygenase-2 (COX-2) was reported [25, 26]. Also, *β*-carotene from other algae *Dunaliella salina (D. salina)* has an improvement potential against liver fibrosis injures induced by thioacetamide (TAA) in rats [19]. In this study, we evaluated the therapeutic effect of *H. pluvialis* extract and its astaxanthin-rich fraction, astaxanthin ester-rich fraction, and *β*-carotene-rich fraction and their mechanisms of action in curing hepatic fibrosis induced by TAA in rats via modulation of MMP and its inhibitor as a target to ameliorate liver fibrosis.

## 2. Materials and Methods

### 2.1. Cultivation of *H. pluvialis*

*H. pluvialis* was isolated from the freshwater community of River Nile water at Cairo, Egypt, in October 2011, and grown on BG11 media [27], which contains NaNO_3_, 1.5 g/l; K_2_HPO_4_, 0.04 g/l; MgSO_4_.7H_2_O, 0.075 g/l; CaCl_2_.7H_2_O, 0.036 g/l; citric acid, 0.006 g/l; Na_2_CO_3_, 0.02 g/l; Na_2_EDTA, 0.001 g/l; ferric ammonium citrate, 0.006 g/l; and 1 ml/l of trace-metal mix A5; A5 contains H_3_BO_3_, 2.86 g/l; MnCl_2_.4H_2_O, 1.81 g/l; ZnSO_4_.7H_2_O, 0.222 g/l; Na_2_ MoO_4_.2H_2_O, 0.39 g/l; CuSO_4_.5H_2_O, 0.079 g/l; and Co(NO_3_)_2_.6H_2_O, 0.0494. Cultivation was carried out in plastic bottles with a capacity of 17 L containing 15 L of BG11 media with continuous aeration. The culture temperature was 22 ± 3°C. Fluorescent light was used to supply constant light intensity ≈2,500 lx for the culture.

After growing for 10 days, the culture was transferred to a fully automated and computer-controlled vertical photobioreactor (Varicon Aqua Solutions Ltd, United Kingdom) with a capacity of 4000 L. Carbon dioxide was injected into the culture, by a gas control unit of the photobioreactor, as a carbon source. The culture was left to grow until the biomass reached 2–2.5 g/l, which is monitored by daily calculation of algal biomass weight (g/l). Algal biomass was harvested by centrifugation at 2000 rpm for 15 min using basket centrifuge. Samples were washed twice with water, dried in an oven at 50°C, ground into a homogenous powder, and stored for further chemical and biological investigation.

### 2.2. Quantification and Identification of *H. pluvialis* Carotenoids

#### 2.2.1. Preparations of Algal Extract and Enrich Fractions

The fine powder of *H. pluvialis* (100 g) was soaked with 1000 ml of dichloromethane: methanol (3 : 1, V/V) in a 2000 ml conical flask and kept on an orbital shaker (Stuart, England) at 160 rpm at room temperature for 24 h. Then, the extract was centrifuged using a centrifuge (Sigma 3-18 ks Centrifuge, Germany) at 5000 rpm for 20 min at 25°C to separate cell debris from the supernatant. The extraction step was repeated twice, and the pooled supernatants were concentrated using a vacuum rotary evaporator (Heidolph Unimax 2010, Germany) at 40°C to dryness giving the crude extract. The crude extract was subjected to a silica gel column chromatography using silica gel, 60-120 *μ*m (Sigma-Aldrich Co., USA), and hexane/ethyl acetate as mobile phase with increasing polarity (0, 10, 30, and100% ethyl acetate) then ethyl acetate: methanol (1 : 1) that afforded 10 fractions that collected in 50 ml per each fraction. The 10 fractions were subjected to TLC (20 × 20 cm aluminum sheets coated with silica gel 60 F254, Merck, Germany) to detect the presence of phytocompounds that were visualized by ultraviolet (UV) fluorescent colors at 254/366 nm UV lamps. Fractions were combined into 3 fractions (1-3) based on TLC results and concentrated to dryness using a rotary evaporator. *β*-Carotene enriches fraction (Fraction 1) and astaxanthin esters enrich fraction (Fraction 2) and astaxanthin enriches fraction (Fraction 3) were confirmed by HPLC. All the used solvents were Analar grade from Sigma-Aldrich Co., USA. All the extraction and column chromatography fractionation steps were performed in dim light.

#### 2.2.2. HPLC Analysis of *β*-Carotene and Astaxanthin

*H. pluvialis* crude extract and beta carotene and astaxanthin enrich fractions were subjected to an Agilent 1260 infinity series HPLC-DAD system (Agilent Technologies, Waldbronn, Germany) equipped with binary gradient Agilent 1260 prep pump (G1361A), an autosampler Agilent 1260 prep ALS (G2260A), and Agilent diode array detector 1260 DAD VL (G1315D) was employed for the detection of the separated *β*-carotene and zeaxanthin. Agilent 5 Prep-C18 Scalar column (5 *μ*m, 150 mm × 4.6 mm) was utilized for separation. The following solvents were used at a flow rate of 1.25 ml/min: (A) acetone and (B) methanol: H2O (9 : 1 *v*/*v*) containing 0.05% BHT. The separation of *β*-carotene and astaxanthin was achieved by a gradient between solvents A and B for 40 min as follows: B was run at 80 to 20% for 25 min, 20% for 10 min, and 20 to 80%for 5 min [28]. The peaks were integrated at 450 nm to quantify *β*-carotene and astaxanthin. *β*-Carotene (C4582-5MG) and all-trans-astaxanthin (SML0982-50MG) were purchased from Sigma-Aldrich Co., USA, and used as standard. *β*-Carotene and all-trans-astaxanthin were identified and quantified by comparing retention time and the peak area of the unknown peak with the *β*-carotene and all-trans-astaxanthin standards. All the used solvents were HPLC grade from Sigma-Aldrich Co., USA.

#### 2.2.3. UHPLC-ESI-MS Analysis

UHPLC-ESI-MS positive ion acquisition mode was carried out on a XEVOTQD triple quadruple instrument, Waters Corporation, Milford, MA01757 U.S.A, mass spectrometer. Mass Lynx™ software version 4.1 (Waters, Milford, MA, USA) was used to control the instruments and for data acquisition and processing. UHPLC chromatographic separations were performed on a reversed-phase column ACQUITYUPLC-BEH C18 (1.7 *μ*m, 2.1 × 50 mm) (Waters, Milford, MA) and a gradient system with the mobile phase consisting of solvent A: acetonitrile: methanol (70 : 30, *v*/*v*) and solvent B: H_2_O 100%. The gradient program used is shown in Table 1 and ESI-mass conditions; polarity (positive), capillary (kV) (3) cone (V) (30), extractor (V) (2), RF (V) (0.5), source temperature (°C) (150), probe temperature (°C) (450), cone gas flow (L/h) (10), desolvation gas flow (L/h) (440), and collision gas flow (mL/min)(0.15), following the methods of [29]. The column was thermostated at 32°C, and the sample temperature was set at 25°C. Before use, all solutions were filtered through 0.2 *μ*m Membrane Nylon White Plain (Millipore, Bedford, MA, USA). Chromatographic peaks were identified by comparing positive ion ESI-MS spectra against known standards or samples. All the used solvents were HPLC grade from Sigma-Aldrich Co., USA.

### 2.3. Liver Fibrosis Experiment

#### 2.3.1. Animals

Adult male albino rats weighing 150-200 g each were purchased from the Animal House at the National Research Centre (NRC, Egypt). Rats were maintained under standard conditions of temperature (25°C) with a 12 h (light)–12 h (dark) cycle and were allowed free access to water and standard laboratory food containing vitamin mixture 1%, mineral mixture 4%, corn oil 10%, sucrose 20%, cellulose 0.2%, casein (95% pure) 10.5%, and starch 54.3% [30]. This study has been approved by the ethics committees of the Committee of Animal Care and Use of NRC (Egypt). All procedures and experiments were performed according to the protocol approved by them, and the animals were treated according to the national and international ethics guidelines.

#### 2.3.2. Chemicals

Thioacetamide (TAA) was purchased from Sigma-Aldrich, USA. Silymarin was obtained from MEPACO, Egypt; all other chemicals, used throughout the experiment, were of the highest analytical grade available.

#### 2.3.3. Experimental Design

After an acclimatization period of one week, rats were randomly allocated into seven groups (8 animals per group), according to the following scheme: Group 1: the normal control group, where rats were injected intraperitoneally with water containing 0.1% Tween 80 twice per week for 6 weeks then received it orally for 4 weeks. Group 2: the fibrotic control (TAA) group, where rats have injected TAA (200 mg/kg, i.p.) twice per week for 6 weeks [31]. Group 3: rats received silymarin (100 mg/kg, orally) [32] daily for 4 weeks after TAA injection. Group 4-7: rats received orally crude extract (200 mg/kg), astaxanthin ester (30 mg/kg), astaxanthin (30 mg/kg), and *β*-carotene (30 mg/kg) [16] daily for 4 weeks after TAA injection.

At the end of the experiment, rats were anesthetized with pentobarbital sodium. Blood samples were withdrawn from the retro-orbital plexus of the rats under the same anesthesia; then, rats were sacrificed by decapitation [33] under the same anesthesia for the collection of liver samples. A 0.5 gm of the liver of each animal was rapidly dissected out, washed, and homogenized using phosphate-buffered saline (PBS, 50 mM potassium phosphate, pH 7.5) at 4°C to produce a 20% homogenate using a homogenizer (Heidolph, DIAX 900, Germany). The homogenates were centrifuged at 2000 × g for 20 min at 4°C then stored at -80°C till the time of analysis [34]. Another part of liver tissues was kept in 10% formalin-saline for histopathological examination.

#### 2.3.4. Assessment of Liver Function Biomarkers

Levels of serum alanine aminotransferase (ALT), aspartate aminotransferase (AST), total bilirubin, and albumin were determined colorimetrically using Biodiagnostic kits, Egypt (CAT. NO: AL 10 31(45), AS 10 61 (45), BR 1111, and AB 10 10).

#### 2.3.5. Assessment of Oxidative Stress Markers

Levels of serum catalase activity and nitric oxide (NO) were determined colorimetrically using Biodiagnostic kits, Egypt (CAT. NO. CA 25 17, NO 25 33).

#### 2.3.6. Assessment of Fibrotic and Antifibrotic Biomarkers

Liver homogenates were assayed for transforming growth factor (TGF-*β*) alpha-smooth muscle actin (*α*-SMA), collagen 1, metalloproteinase-9 (MMP9), and tissue inhibitors of metalloproteinase-1 (TIMP-1) using SinoGeneClon Biotech Co., Ltd, ELISA kits (CAT. NO. SG-20557, SG-20946, SG-20412, SG-20877).

#### 2.3.7. Assessment of Proinflammatory Biomarkers

Tumor necrosis factor-alpha (TNF-*α*) and interleukin 6 (IL-6) were determined using specific Rat ELISA kits of Elabscience, China (CAT.No.E-EL-R0019) and Sunlong Biotech Co., Ltd, China (CAT. No. SL0411Ra).

#### 2.3.8. Histological Examination

For histopathologic assessment, the parts of the livers were fixed in 10% formalin solution then dehydrated in ascending grades of alcohol and embedded in paraffin. Four sections/group, at 4 *μ*m thickness, were taken and stained with hematoxylin and eosin (H&E). The severity of histopathological alternation was semiquantitatively assessed based on liver histology evaluated by a blinded pathologist using a scoring system in which score 0 indicated no alternation; score 1, mild alternation; score 2, alternation activity; and score 3, severe alternation.

### 2.4. Statistical Analysis

All the values are presented as means ± standard error of the means (SE). Data were evaluated by one-way analysis of variance followed by Fisher's LSD comparisons test. GraphPad Prism software, version 5 (Inc., San Diego, USA) was used to carry out these statistical tests. The difference was considered significant when *P* < 0.05.

## 3. Results

### 3.1. Quantification and Identification of *H. pluvialis* Carotenoids

The extraction of fine powder of *H. pluvialis* with dichloromethane: methanol (3 : 1, *V*/*V*) revealed crude extract with an extraction yield (6.1%) containing *β*-carotene (12.95 mg/g, extract) and all-trans-astaxanthin (10.85 mg/g, extract) as quantified by HPLC and presented in Figure 1. The silica column chromatography fractionation proved 3 main fractions based on HPLC analysis; *β*-carotene enriches fraction (Fraction 1) containing 77% beta-carotene (Figure 2) equivalent to 77.56 mg/g of *β*-carotene enriches fraction, astaxanthin esters enriches fraction (Fraction 2) containing mono and di-esters of free astaxanthin (Figure 3), and astaxanthin enriches fraction (Fraction 3) containing 27.9% all-trans-astaxanthin (Figure 4) equivalent to 16.21 mg/g of astaxanthin enriches fraction.

Figure 5 displays the UHPLC/ESI-MS chromatogram in the positive ion of crude extract of *H. pluvialis*, the results of carotenoids analysis leads to the identification of 28 carotenoids based on their molecular ion [M]^+^, protonated quasimolecular ion [M + H]^+,^ and alkaline metal adduct ions [M + Na]^+^ and [M + K]^+^ as presented in Table 2. The m/z 593 and 616, and 632 are assumed to be [M]^+.^, [M + Na]^+^, and [M + K]^+^ of astaxanthin (Figure 6(a)). The m/z 635 and 558 are assumed to be [M]^+.^ and [M + Na]^+^ of *α* or *β*-carotene(Figure 6(b)). The m/z 568, 569, and 476 are assumed to be [M]^+.^, [M + H]^+^, and [M-92] of lutein or zeaxanthin (Figure 6(c)). Regarding the astaxanthin monoester, there are 14 peaks that were identified as astaxanthin monoester such as the m/z 932 is assumed to be [M + NA]^+^ of astaxanthin monoester- C22:4 (Figure 6(d)). While 5 peaks were identified as astaxanthin diester, the m/z 953 is assumed to be [M + H]^+^ of astaxanthin diester-C16:4/C8:0 (Figure 6(e)).

### 3.2. Liver Fibrosis

#### 3.2.1. Effects of *H. pluvialis* Crude Extract and Its Fractions (Astaxanthin, Astaxanthin Ester, and *β*-Carotene) on Serum Hepatic Function Biomarkers

Injection of TAA, for 6 weeks, led to a significant elevation in ALT and AST activities as well as total bilirubin serum level with a decrease in albumin serum level compared to those in the control rats. Treatment with silymarin, for 4 weeks, resulted in a significant decrease in serum level of ALT, AST, and total bilirubin with an increase in albumin serum level as compared to the TAA group. Administration of *H. pluvialis* crude extract and its fractions (astaxanthin, astaxanthin ester, and *β*-carotene) for 4 weeks reduced serum levels of ALT, AST, and total bilirubin with an increase in albumin serum level as compared to the TAA group. Moreover, crude extract-treated rats showed a decrease in serum level of ALT and AST by 10% and 17%, respectively, as compared to the silymarin group, returning the serum liver biomarkers to their normal values (Table 3).

#### 3.2.2. Effects of *H. pluvialis* Crude Extract and Its Fractions (Astaxanthin, Astaxanthin Ester, and *β*-Carotene) on Oxidative Stress Biomarkers

Serum catalase activity was decreased, and NO level was elevated with TAA injection as compared to normal group values. On the other hand, treatment with silymarin, for 4 weeks, resulted in a significant increase in serum activity of catalase with a significant decrease in NO serum level, as compared to the TAA group. Treatment with *H. pluvialis* crude extract and its fractions (astaxanthin, astaxanthin ester, and *β*-carotene) for 4 weeks resulted in an elevation in catalase activity with a decrease in NO level, as compared to the TAA group. Treatment with crude extract showed an increase in catalase activity with a decline in NO level by 28% and 9%, respectively, as compared to the silymarin group, returning the serum levels of catalase and NO to their normal values (Table 4).

#### 3.2.3. Effects of *H. pluvialis* Crude Extract and Its Fractions (Astaxanthin, Astaxanthin Ester, and *β*-Carotene) on Fibrotic and Antifibrotic Biomarkers

Induction of liver fibrosis in rats using TAA for 6 weeks resulted in a significant elevation in hepatic contents of TGF-*β*1, *α*-SMA, collagen 1, and TIMP1 and reduced MMP9 content as compared to the normal group. Treatment with silymarin, for 4 weeks, reduced hepatic contents of TGF-*β*1, *α*-SMA, collagen 1, and TIMP1 and elevated MMP9 content as compared to the TAA group. Moreover, treatment with *H. pluvialis* crude extract and its fractions (astaxanthin, astaxanthin ester, and *β*-carotene) for 4 weeks significantly decreased the raised hepatic TGF-*β*1, *α*-SMA, collagen1, and TIMP1 contents and elevated MMP9 content as compared to the TAA group. Treatment with crude extract showed a decrease in hepatic contents of TGF-*β*1, collagen 1, and TIMP1 and elevated MMP9 content by 78%, 35%, 17%, and 13%, respectively, as compared to the silymarin group. Treatment with crude extract returned hepatic contents of TGF-*β*1, *α*-SMA, collagen 1, TIMP1, and MMP9 to their normal values (Figure 7).

#### 3.2.4. Effects of *H. pluvialis* Crude Extract and Its Fractions (Astaxanthin, Astaxanthin Ester, and *β*-Carotene) on Proinflammatory Cytokine Biomarkers

Induction of liver fibrosis in rats using TAA for 6 weeks resulted in a significant elevation in hepatic contents of IL-6 and TNF-*α*, as compared to the normal group. Treatment with silymarin, for 4 weeks, reduced hepatic contents of IL-6 and TNF-*α* as compared to the TAA group. Moreover, treatment with *H. pluvialis* crude extract and its fractions (astaxanthin, astaxanthin ester, and *β*-carotene) for 4 weeks significantly decreased the elevated hepatic IL-6 and TNF-*α* as comparing to the TAA group. Treatment with crude extract showed a decrease in hepatic contents IL-6 and TNF-*α* by 39% and 31%, respectively, as compared to the silymarin group. Treatment with crude extract returned hepatic contents of IL-6 and TNF-*α* to their normal values (Figure 8).

#### 3.2.5. Histopathological Findings

Figure 9 summarised the effects of *H. pluvialis* crude extract and its fractions (astaxanthin, astaxanthin ester, and *β*-carotene) on histopathological alteration.

The liver section of the control normal rat showed no histopathological alteration, and the normal histological structure of the central vein and surrounding hepatocytes in the parenchyma was recorded (Figure 10(a)). The liver section of the TAA-treated group that showed fine fibroblastic cell proliferation was dividing the degenerated and necrobiotic changes hepatocytes into lobules (Figure 10(b)). Liver section of the silymarin-treated group there was few pigmented cells infiltration surrounding and adjacent to the dilated central vein (Figure 10(c)). The liver section of the crude extract showed diffuse Kupffer cell proliferation was detected in between the degenerated hepatocytes (Figure 10(d)). The liver section of astaxanthin ester showed Kupffer cell proliferation was detected in between the hepatocytes (Figure 10(e)). The liver section of astaxanthin showed mild degeneration in the hepatocytes adjacent to the congested central vein. A focal hemorrhage was detected in the parenchyma adjacent to the portal area (Figure 10(f)). The liver section of *β*-carotene showed dilatation in the central vein associated with focal hemorrhage in the parenchyma. Fine fibroblastic cell proliferation was dividing the degenerated and necrobiotic changed hepatocytes into lobules (Figure 10(g)).

The liver section of the portal area of the TAA-treated group showed fibrosis with inflammatory cell proliferation between the congested portal vein and hyperplastic bile ducts (Figure 11(a)). In the liver section of the silymarin-treated group, the portal area showed inflammatory cell infiltration (Figure 11(b)). The liver section of crude extract in the portal area showed few inflammatory cell infiltration (Figure 11(c)). Liver section of astaxanthin ester associated with inflammatory cells infiltration in the portal area (Figure 11(d)). The liver section of astaxanthin showed a focal hemorrhage detected in the parenchyma adjacent to the portal area (Figure 11(e)). The liver section of *β*-carotene the portal area showed congestion in the portal vein and mild fibrosis with inflammatory cell infiltration in between (Figure 11(f)).

## 4. Discussion

The HPLC analysis of *H. pluvialis* carotenoid extract showed the presence of free astaxanthin and *β*-carotene based on the available standers; these results agree with [21]. Because the main crude extract and astaxanthin ester rich fraction showed the potent effects against liver fibrosis as compared with astaxanthin and *β*carotene-rich fractions, so the individual components in the crude extract were analyzed by LC/ESI-MS in the positive-ion mode. The ESI-MS chromatogram presumed the identification of several carotenoids in the crude extract of *H. pluvialis* including three isomers of astaxanthin, *α* or *β*-carotene, lutein or zeaxanthin, 9′-cis-neoxanthin, and *β*-cryptoxanthin, plus several astaxanthin mono and di-esters; these results are in accord with the results of [35, 36]. In these results, the ESI-MS of astaxanthin provides molecular ion [M]^+^ predominantly along with alkaline metal adduct ions [M + Na]^+^ and [M + K]^+^ at m/z 593 and 616, and 632. While in other studies, the ESI-MS of astaxanthin provides the protonated quasimolecular ions [M + H]^+^ at m/z 597 [35, 36]. The ESI-MS of lutein or zeaxanthin in this result provides molecular ion [M]^+^ and protonated quasimolecular ions [M + H]^+^ at m/z 568 and 569; this is in accord with [29, 36]. The ESI-MS of *α* or *β*-carotene provides molecular ion [M]^+^ and alkaline metal adduct ion [M + Na]^+^ at m/z 535 and 558; this result is in accord with [29]. The ESI-MS of different astaxanthin mono and di-esters in this study provides protonated quasimolecular ions [M + H]^+^ and alkaline metal adduct ion [M + Na]^+^, such as astaxanthin monoester-C22:6 provides [M + NA]^+^ at m/z 929, as previously reported by [37], astaxanthin monoester-C22:4 provides [M + NA]^+^ at m/z 932, while astaxanthin monoester-C16:4 provides [M + H]^+^ at m/z 828, as previously reported by [36]. The *H. pluvialis* contains astaxanthin diester-C16:4/C8:0 provides [M + H]^+^ at m/z 953, and astaxanthin diester-C16:1/C11:0 provides [M + Na]^+^ at m/z 983. The potent activity of crude extract and astaxanthin ester-rich fraction of *H. pluvialis* against liver fibrosis in this study might be thanks to the association of astaxanthin with different fatty acids that increase the bioavailability of astaxanthin in different tissues accordingly increases its bioactivity [38].

Liver fibrosis is closely related to oxidative stress. As previously mentioned, TAA induced oxidative stress, hepatocellular fibrosis, and necrosis [32], overexpressed the iNOS gene, and produced apoptotic DNA fragmentation [39]. Antioxidants have a protective effect in animal models and clinical trials on liver fibrosis [40]. In the current study, the potent competency of different carotenoid individuals including astaxanthin and *β*-carotene is their ameliorative ability against oxidative stress in liver diseases. TAA increased ALT, AST, and total bilirubin serum levels with a reduction in albumin serum level as shown in a previous study [41], however, administration of *H. pluvialis* crude extract and its fractions (astaxanthin, astaxanthin ester, and *β*-carotene) effectively reduced liver function with an increase in albumin serum level. Only the administration of *H. pluvialis* crude extract returned the serum levels of ALT, AST, total bilirubin, and albumin to their normal levels. In these contexts, the *H. pluvialis* carotenoids alleviated doxorubicin-induced liver injury through decreasing liver function and regulating Keap1/Nrf2/HO-1 pathway [42]. Also, the liver is more vulnerable to TAA-induced liver oxidative damage evidenced by higher NO serum level and lower catalase activity, while all treatments especially crude extract have antioxidant effects as confirmed by the detection of oxidant and antioxidant indicators as NO serum level and catalase activity. The administration of *H. pluvialis* crude extract and its fractions (astaxanthin, astaxanthin ester, and *β*-carotene) effectively reduced the liver oxidative damage and inflammation induced by TAA administration in this study, especially the administration of *H. pluvialis* crude extract returning the levels of NO, CAT, IL-6, and TNF-*α* to its normal levels, this might be thanks to the potent antioxidant activity of the different carotenoids including astaxanthin and *β*-carotene identified in *H. pluvialis* crude extract by LC/ESI-MS. The administration of *H. pluvialis* carotenoids astaxanthin enhanced the levels of SOD and CAT and decreased the lipid peroxidation against liver injury induced by doxorubicin in rats [42]. Also, *β*-carotene, from other algae *D. Saline*, exerted its antioxidant through inducing catalase and thioredoxin enzymes that attenuated STZ-induced diabetic neuropathy [43] and elevated the levels of GSH with a decrease in MDA opposing hepatic fibrosis induced by TAA in rats [44]. *β*-Cryptoxanthin, one of the other carotenoids, found in our crude extract has an antioxidant effect against oxidative DNA damage and lipid peroxidation [45]. Moreover, it has anti-inflammatory activity modulating macrophage immune response [46]. This carotenoid suppressed proinflammatory cytokines secretion (TNF-*α* and IL-6) [46] reversing inflammation, steatosis, and fibrosis progression in NASH by repressed macrophage activation [47]. In patients with nonalcoholic fatty liver disease (NAFLD), *β*-cryptoxanthin intake elevated antioxidant and anti-inflammatory effects [15]. Lutein is one of the natural *H. pluvialis* carotenoids; its supplementation alleviated hepatic lipid accumulation, preventing NAFLD induced by a high-fat diet [48].

HSCs, collagen-producing cells, contribute to ECM deposition [49] and have a pivotal role in liver fibrosis [50]. Our results explored that TAA expressed TGF-*β* activating HSCs and increased liver contents of *α*-SMA and collagen 1, while *H. pluvialis* crude extract and its fractions (astaxanthin, astaxanthin ester, and *β*-carotene) suppressed the activation of HSCs, inhibited profibrotic gene expression via preventing the release of TGF-*β*, and decreased liver contents of *α*-SMA and collagen 1. Especially, astaxanthin ester has a direct method of preventing and treating liver fibrosis through reducing the activation of HSCs and decreasing ECM components and deposition that evidenced in this study by decreased liver contents of collagen-1 and *α*-SMA. Further evidence has shown that astaxanthin (80 mg/kg), during liver fibrosis, inhibited the expression of TGF-*β* and activation of HSCs [51, 52]. Also, *β*-carotene from *D. salina* treating liver fibrosis via decrement of *α*-SMA and COL-1 liver contents [19].

MMPs, in fibrosis, can degrade ECM protein components and promote activated HSC apoptosis [53]. This current study is the first to explore the effects of crude extract and its carotenoid enrich fractions on liver fibrosis induced by TAA via increasing MMP9 and decreasing its inhibitor TIMP1expression. Some molecules become stimulated as MMPs during liver fibrosis restoration, and other molecules become repressed as MMP inhibitor. Our results exhibited that crude extract and its carotenoid enrich fractions play a dual role in liver fibrosis as preserved the balance between MMP9/TIMP1 ameliorating liver fibrosis. These results were simultaneously confirmed in a histopathological study that showed amelioration of liver fibrosis and inflammatory cell proliferation in all treatment groups, especially crude extract. These results might be owing to the presence of the potent antioxidant carotenoids (astaxanthin and *β*-carotene) in the used extract of *H. pluvialis*; these results are in accord with other studies that confirmed the antifibrotic effect of astaxanthin in the CCL4 model of liver fibrosis [54]. The antifibrotic effect of *β*-carotene of *D. salina* through the inhibition of the TGF-*β* expression and increasing MMP9 was also reported previously [55].

Kupffer cell is a sensor for tissue integrity and homeostasis in the liver and functions as a primary defense line against invading microorganisms and maintaining immunological tolerance and providing an anti-inflammatory in the liver and in [56]. For instance, it secretes interleukin-10, the anti-inflammatory cytokine [57]. Crude extract and its carotenoid enrich fractions in this study, for the first time, increased the number of Kupffer cells, as shown in the current histopathological study, that expressed MMP9, downregulated inflammation, and mediated fibrosis restoration. These results provide a new prospect for treating liver fibrosis, apoptosis, and necrobiosis induced by TAA.

## 5. Conclusion

This study elucidated the therapeutic effect of *H. pluvialis* crude extract and its fractions (astaxanthin, astaxanthin ester, and *β*-carotene) in treating hepatic fibrosis via decreasing ECM components and its deposition, regulating oxidative stress and MMP9/TIMP1 as well as finally activating Kupffer cell. Also, this study showed the mechanisms responsible for the hepatic fibrosis process, increasing interest concerning the translation of *H. pluvialis* and its carotenoid enrich fractions into clinical applications in the future.

## Figures and Tables

**Figure 1:** HPLC analysis of all-trans-astaxanthin and *β*-carotene in *H. pluvialis* dichloromethane: methanol (3 : 1, *V*/*V*) crude extract.

**Figure 2:** HPLC analysis of *β*-carotene in *β*-carotene enriches fraction of *H. pluvialis*.

**Figure 3:** HPLC analysis of astaxanthin esters in astaxanthin esters enriches fraction of *H. pluvialis.*

**Figure 4:** HPLC analysis of all-trans-astaxanthin in astaxanthin enriches fraction of *H. pluvialis.*

**Figure 5:** LC/ESI-MS chromatogram in the positive-ion of crude extract of *H. pluvialis*.

**Figure 6:** ESI-MS positive-ion spectra of (a) astaxanthin, (b) *α* or *β*-carotene, (c) lutein or zeaxanthin, (d) astaxanthin monoester, C22:4, and (e) astaxanthin diester, C16:4/C8:0.

**Figure 7:** Effects of crude extract and its fractions (astaxanthin, astaxanthin ester, and *β*-carotene) on hepatic contents of (a) TGF-*β*, (b) SMA-*α*, (c) collagen 1, (d) TIMP-1, and (e) MMP9. Data are presented as the mean ± S.E. of (*n* = 8) for each group. Statistical analysis was carried out by one-way analysis of variance followed by Fisher's LSD comparisons test. A Statistically significant from the control group. B Statistically significant from the TAA group. C Statistically significant from the silymarin group. D Statistically significant from the crude extract group. E Statistically significant from the astaxanthin ester group at *P* < 0.05.

**Figure 8:** Effects of crude extract and its fractions (astaxanthin, astaxanthin ester, and *β*-carotene) on hepatic contents of (a) IL-6 and (b) TNF-*α*. Data are presented as the mean ± S.E. of (*n* = 8) for each group. Statistical analysis was carried out by one-way analysis of variance followed by Fisher's LSD comparisons test. A Statistically significant from the control group. B Statistically significant from the TAA group. C Statistically significant from the silymarin group. D Statistically significant from the crude extract group. E Statistically significant from the astaxanthin ester group at *P* < 0.05.

**Figure 9:** Effects of crude extract and its fractions (astaxanthin, astaxanthin ester, and *β*-carotene) on histopathological alteration. Data are presented as the mean ± S.E. of (*n* = 8) for each group. Statistical analysis was carried out by one-way analysis of variance followed by Fisher's LSD comparisons test. A Statistically significant from the control group. B Statistically significant from the TAA group. C Statistically significant from the silymarin group. D Statistically significant from the crude extract group. E Statistically significant from the astaxanthin ester group at *P* < 0.05.

**Figure 10:** Liver section of the central vein and surrounding hepatocytes. (a) Liver section of the rat from the control normal rat showed no histopathological alteration and the normal histological structure of the central vein and surrounding hepatocytes in the parenchyma were recorded. (b) Liver section of rats from the TAA-treated group showed fine fibroblastic cell proliferation was dividing the degenerated and necrobiotic changes hepatocytes into lobules. (c) Liver section of rat from the silymarin-treated group there was few pigmented cell infiltration surrounding and adjacent to the dilated central vein (H&E X 400). (d) Liver section of rats from crude extract showed diffuse Kupffer cell proliferation was detected in between the degenerated hepatocytes. (e) Liver section of rats from astaxanthin ester showed Kupffer cell proliferation was detected in between the hepatocytes. (f) Liver section of the rat from astaxanthin showed degeneration in the hepatocytes adjacent to the congested central vein. (g) Liver section of rats from *β*-carotene showed dilatation in the central vein associated with focal hemorrhage in the parenchyma. Fine fibroblastic cell proliferation was dividing the degenerated and necrobiotic changed hepatocytes into lobules. (H&E X 400 bar scale: 50 *μ*m).

**Figure 11:** Liver sections of the portal area. (a) Liver section of the portal area of rats from the TAA-treated group showed fibrosis with inflammatory cell proliferation in between the congested portal vein and hyperplastic bile ducts. (b) Liver section of rats from the silymarin-treated group of the portal area showed inflammatory cell infiltration. (c) Liver section of the rat from crude extract showed the portal area showed few inflammatory cell infiltration. (d) Liver section of the rat from the astaxanthin ester showed inflammatory cell infiltration in the portal area. (e) Liver section of rat from astaxanthin focal hemorrhage was detected in the parenchyma adjacent to the portal area. (f) Liver section of rats from *β*-carotene of the portal area showed congestion in the portal vein and mild fibrosis with inflammatory cell infiltration in between. (H&E X 400 bar scale:50 *μ*m).

**Table 1:** Gradient profile used in the chromatographic separation of carotenoids.

Time (min)	Flow rate (ml/min)	A (%, *v*/*v*)	B (%, *v*/*v*)	Curve
Initial	0.4	85	15	Linear
2.0	0.4	85	15	Linear
3.0	0.4	100	0	Linear
7.0	0.4	100	0	Linear
8.0	0.6	100	0	Linear
11.6	0.6	100	0	Linear
12.6	0.4	85	15	Linear
15.0	0.4	85	15	Linear

**Table 2:** Identified carotenoids especially astaxanthin esters in *H. pluvialis* by LC/ESI-MS.

No.	Peake Rt (min).	m/z	Compound
1	1.80	625 [M + Na]^+^	9′-cis-Neoxanthin
2	1.97	593 [M] + ., 616 [M + Na]^+^, and 633 [M + K]^+^	Astaxanthin (isomer 1)
3	2.02	633 [M + K]^+^	Astaxanthin (isomer 2)
4	2.20	633 [M + K]^+^	Astaxanthin (isomer 2)
5	2.65	558 [M + Na]^+^	*α* or *β*-carotene
6	2.89	568 [M] + ., 569[M + H]^+^	Lutein or Zeaxanthin
7	3.01	645 [M + Na]^+^	Adonirubin acetate
8	3.39	455 [M + K]^+^	*β*-Apo-8′-carotenal
9	3.67	929 [M + NA]^+^	Astaxanthin monoester, C22:6
10	3.73	575 [M + Na]^+^	*β*-Cryptoxanthin
11	3.98	828 [M + H]^+^	Astaxanthin monoester, C16:4 (isomer 1)
12	4.04	932 [M + Na]^+^	Astaxanthin monoester, C22:4
13	4.18	934 [M + Na]^+^	Astaxanthin monoester, C22:3 (isomer 1)
14	4.30	828 [M + H]^+^	Astaxanthin monoester, C16:4 (isomer 2)
15	4.32	934 [M + Na]^+^	Astaxanthin monoester, C22:3 (isomer 2)
16	4.39	745 [M + Na]^+^	Astaxanthin monoester, C8:0
17	4.46	953 [M + H]^+^	Astaxanthin diester, C16:4/C8:0 (isomer 1)
18	4.56	830 [M + H]^+^	Astaxanthin monoester, C16:3
19	4.72	832 [M + H]^+^	Astaxanthin monoester, C16:2
20	4.75	912 [M + Na]^+^	Astaxanthin monoester, C20:1 (isomer 1)
21	4.90	938 [M + Na]^+^	Astaxanthin monoester, C22:2
22	5.09	983 [M + Na]^+^	Astaxanthin diester, C16:1/C11:0
23	5.19	940 [M + Na]^+^	Astaxanthin monoester, C22:1
24	5.41	953 [M + H]^+^	Astaxanthin diester, C16:4/C8:0 (isomer 2)
25	5.69	942 [M + Na]^+^	Astaxanthin monoester, C22:0
26	6.57	976 [M + Na]^+^	Astaxanthin diester, C16:4/C8:0
27	6.62	971 [M + Na]^+^	Astaxanthin diester, C12:0/C11:0
28	7.98	912 [M + Na]^+^	Astaxanthin monoester, C20:1 (isomer 2)

**Table 3:** Effects of *H. pluvialis* crude extract and its fractions (astaxanthin, astaxanthin ester, and *β*-carotene) on serum hepatic functions biomarkers.

	Normal control	TAA	Silymarin (100 mg/kg)	Crude extract (200 mg/kg)	Astaxanthin ester (30 mg/kg)	Astaxanthin (30 mg/kg)	*Β*-carotene (30 mg/kg)
ALT (U/L)	73.59 ± 0.8	107.7 ± 3.6^a^	84.8 ± 2.6^ab^	76.6 ± 2.6^bc^	82.71 ± 1.3^ab^	86.7 ± 2.4^abd^	90.2 ± 1.8^abde^
(% of TAA control)			79%	71%	77%	81%	84%
AST (U/L)	82.33 ± 7.4	171 ± 7.9^a^	101.9 ± 5.2^ab^	83.58 ± 3.8^bc^	102.7 ± 1.4^abd^	107.7 ± 2.7^abd^	108.3 ± 3^abd^
(% of TAA control)			60%	49%	60%	63%	63%
Bilirubin (mg/dl)	4.78 ± 0.05	8.68 ± 0.28^a^	5.25 ± 0.05^b^	5 ± 0.28^b^	5.67 ± 0.5^ab^	7.53 ± 0.22^abcde^	7.88 ± 0.2^abcde^
(% of TAA control)			60%	58%	65%	87%	91%
Albumin (g/dl)	4.29 ± 0.43	2.16 ± 0.01^a^	3.83 ± 0.04^b^	4.01 ± 0.02^b^	3.8 ± 0.06^ab^	2.77 ± 0.01^abcde^	2.63 ± 0.02^abcde^
(% of TAA control)			177%	186%	176%	128%	122%

Data are presented as the mean ± S.E. of (*n* = 8) for each group and % of the TAA group. Statistical analysis was carried out by one-way analysis of variance followed by Fisher's LSD comparisons test. ^a^Statistically significant from the control group. ^b^Statistically significant from the TAA group. ^c^Statistically significant from the silymarin group. ^d^Statistically significant from crude extract group. ^e^Statistically significant from Astaxanthin ester group at *P* < 0.05.

**Table 4:** Effects of *H. pluvialis* crude extract and its fractions (astaxanthin, astaxanthin ester, and *β*-carotene) on serum levels of oxidative stress biomarkers.

	Normal control	TAA	Silymarin (100 mg/kg)	Crude extract (200 mg/kg)	Astaxanthin ester (30 mg/kg)	Astaxanthin (30 mg/kg)	*β*-Carotene (30 mg/kg)
Catalase (U/L)	357.3 ± 9.6	106.4 ± 8.3^a^	250 ± 19.33^ab^	318.8 ± 29.8^bc^	278.7 ± 17.2^ab^	247 ± 20.7^abd^	219.25 ± 16.1^abde^
(% of TAA control)			235%	300%	262%	233%	206%
NO (*μ*mol/L)	48.25 ± 0.37	80.93 ± 2.11^a^	57.25 ± 0.29^ab^	51.9 ± 2.17^bc^	53 ± 1.12^ab^	53.52 ± 0.93^ab^	61.17 ± 0.39^abde^
(% of TAA control)			71%	64%	66%	66%	76%

Data are presented as the mean ± S.E. of (*n* = 8) for each group and % of the TAA group. Statistical analysis was carried out by one-way analysis of variance followed by Fisher's LSD comparisons test. ^a^Statistically significant from the control group. ^b^Statistically significant from the TAA group. ^c^Statistically significant from the silymarin group. ^d^Statistically significant from crude extract group. ^e^Statistically significant from astaxanthin ester group at *P* < 0.05.

## Data Availability

Data are available with the corresponding author.

## References

[1] Campana L., Iredale J. P. (2017). Regression of liver fibrosis. *Seminars in liver disease*.

[2] Befeler A. S., Di Bisceglie A. M. (2002). Hepatocellular carcinoma: diagnosis and treatment. *Gastroenterology*.

[3] El-Serag H. B. (2002). Hepatocellular carcinoma and hepatitis C in the United States. *Hepatology*.

[4] Pinzani M., Rombouts K., Colagrande S. (2005). Fibrosis in chronic liver diseases: diagnosis and management. *Journal of Hepatology*.

[5] Baghy K., Iozzo R. V., Kovalszky I. (2012). Decorin–TGF*β* axis in hepatic fibrosis and cirrhosis. *Journal of Histochemistry & Cytochemistry*.

[6] Fallowfield J. A., Mizuno M., Kendall T. J. (2007). Scar-associated macrophages are a major source of hepatic matrix metalloproteinase-13 and facilitate the resolution of murine hepatic fibrosis. *The Journal of Immunology*.

[7] Feng M., Ding J., Wang M., Zhang J., Zhu X., Guan W. (2018). Kupffer-derived matrix metalloproteinase-9 contributes to liver fibrosis resolution. *International Journal of Biological Sciences*.

[8] Aoyama T., Kuwahara-Arai K., Uchiyama A. (2017). Spleen-derived lipocalin-2 in the portal vein regulates Kupffer cells activation and attenuates the development of liver fibrosis in mice. *Laboratory Investigation*.

[9] Lu L., Feng M., Gu J. (2013). Restoration of intrahepatic regulatory T cells through MMP-9/13-dependent activation of TGF-*β* is critical for immune homeostasis following acute liver injury. *Journal of Molecular Cell Biology*.

[10] Ramachandran P., Pellicoro A., Vernon M. A. (2012). Differential Ly-6C expression identifies the recruited macrophage phenotype, which orchestrates the regression of murine liver fibrosis. *Proceedings of the National Academy of Sciences*.

[11] Bi W.-R., Yang C.-Q., Shi Q. (2012). Transforming growth factor-*β*1 induced epithelial-mesenchymal transition in hepatic fibrosis. *Hepato-Gastroenterology*.

[12] Arthur M. J. (2000). Fibrogenesis II. Metalloproteinases and their inhibitors in liver fibrosis. *American Journal of Physiology-Gastrointestinal and Liver Physiology*.

[13] Sentíes-Gómez M. D., Gálvez-Gastélum F. J., Meza-García E., Armendáriz-Borunda J. (2005). Hepatic fibrosis: role of matrix metalloproteases and TGFbeta. *Gaceta Médica de México*.

[14] Bonet M. L., Canas J. A., Ribot J., Palou A. (2016). Carotenoids in adipose tissue biology and obesity. *Carotenoids in Nature*.

[15] Elvira-Torales L. I., García-Alonso J., Periago-Castón M. J. (2019). Nutritional importance of carotenoids and their effect on liver health: a review. *Antioxidants*.

[16] El-Baz F. K., Hussein R. A., Jaleel G. A. R. A., Saleh D. O. (2018). Astaxanthin-rich *haematococcus pluvialis* algal hepatic modulation in D-galactose-induced aging in rats: role of Nrf2. *Advanced pharmaceutical bulletin*.

[17] Fiedor J., Burda K. (2014). Potential role of carotenoids as antioxidants in human health and disease. *Nutrients*.

[18] Ali S. I., Gaafar A. A., Abdallah A. A., El-Daly S. M., El-Bana M., Hussein J. (2018). Mitigation of alpha-cypermethrin-induced hepatotoxicity in rats by Tribulus terrestris rich in antioxidant compounds. *Jordan Journal of Biological Sciences*.

[19] El-Baz F. K., Ali S. I., Basha M. (2020). Design and evaluation of bioenhanced oral tablets of *Dunaliella salina* microalgae for treatment of liver fibrosis. *Journal of Drug Delivery Science and Technology*.

[20] Bolhassani A. (2015). Cancer chemoprevention by natural carotenoids as an efficient strategy. *Anti-Cancer Agents in Medicinal Chemistry (Formerly Current Medicinal Chemistry-Anti-Cancer Agents)*.

[21] Kamath B. S., Srikanta B. M., Dharmesh S. M., Sarada R., Ravishankar G. A. (2008). Ulcer preventive and antioxidative properties of astaxanthin from _*Haematococcus pluvialis*_. *European Journal of Pharmacology*.

[22] Masoudi A., Dargahi L., Abbaszadeh F. (2017). Neuroprotective effects of astaxanthin in a rat model of spinal cord injury. *Behavioural Brain Research*.

[23] Wang X., Zhao H., Shao Y. (2014). Nephroprotective effect of astaxanthin against trivalent inorganic arsenic-induced renal injury in Wistar rats. *Nutrition Research and Practice*.

[24] Christen W. G., Gaziano J. M., Hennekens C. H., PHYSICIANS FT, STUDY II HE (2000). Design of Physicians' Health Study II—a randomized trial of beta-carotene, vitamins E and C, and multivitamins, in prevention of cancer, cardiovascular disease, and eye disease, and review of results of completed trials. *Annals of Epidemiology*.

[25] Bai S.-K., Lee S.-J., Na H.-J. (2005). *β*-Carotene inhibits inflammatory gene expression in lipopolysaccharide- stimulated macrophages by suppressing redox-based NF-*κ*B activation. *Experimental & Molecular Medicine*.

[26] Hadad N., Levy R. (2012). The synergistic anti-inflammatory effects of lycopene, lutein, *β*-carotene, and carnosic acid combinations via redox-based inhibition of NF-*κ*B signaling. *Free Radical Biology and Medicine*.

[27] Abdo S. M., Ahmed E., El-Enin S. A., El Din R. S., El Diwani G., Ali G. (2013). Growth rate and fatty acids profile of 19 microalgal strains isolated from river Nile for biodiesel production. *Journal of Algal Biomass Utilization*.

[28] Sarada R., Vidhyavathi R., Usha D., Ravishankar G. (2006). An efficient method for extraction of astaxanthin from green alga *Haematococcus pluvialis*. *Journal of Agricultural and Food Chemistry*.

[29] Rivera S., Vilaró F., Canela R. (2011). Determination of carotenoids by liquid chromatography/mass spectrometry: effect of several dopants. *Analytical and Bioanalytical Chemistry*.

[30] Salama A. A. A., Ibrahim B. M. M. (2015). Neurotherapeutic effect of allopurinol against brain injury in hyperlipidemic rats. *African Journal of Pharmacy and Pharmacology*.

[31] Liu Y.-W., Chiu Y.-T., Fu S.-L., Huang Y.-T. (2015). Osthole ameliorates hepatic fibrosis and inhibits hepatic stellate cell activation. *Journal of Biomedical Science*.

[32] Mansour H. M., Salama A. A. A., Abdel-Salam R. M., Ahmed N. A., Yassen N. N., Zaki H. F. (2018). The anti-inflammatory and anti-fibrotic effects of tadalafil in thioacetamide-induced liver fibrosis in rats. *Canadian Journal of Physiology and Pharmacology*.

[33] Salama A., Hegazy R., Hassan A. (2016). Intranasal chromium induces acute brain and lung injuries in rats: assessment of different potential hazardous effects of environmental and occupational exposure to chromium and introduction of a novel pharmacological and toxicological animal model. *PLoS One*.

[34] Salama A. A., Zaki H. F., Siham M., EL-Denshary E., Ismaiel I. E.-K. (2015). Antiasthmatic effects of evening primrose oil in ovalbumin-allergic rats. *Der Pharmacia Lettre*.

[35] Miao F., Lu D., Li Y., Zeng M. (2006). Characterization of astaxanthin esters in _*Haematococcus pluvialis*_ by liquid chromatography -atmospheric pressure chemical ionization mass spectrometry. *Analytical Biochemistry*.

[36] Weesepoel Y., Vincken J. P., Pop R. M., Liu K., Gruppen H. (2013). Sodiation as a tool for enhancing the diagnostic value of MALDI-TOF/TOF-MS spectra of complex astaxanthin ester mixtures from *Haematococcus pluvialis*. *Journal of Mass Spectrometry*.

[37] Frassanito R., Flaim G., Mancini I., Guella G. (2006). High production of unexpected carotenoids in Dinophyceae. Astaxanthin esters from the freshwater dinoflagellate _*Tovellia sanguinea*_. *Biochemical Systematics and Ecology*.

[38] de Carvalho C. C. C. R., Caramujo M. J. (2017). Carotenoids in aquatic ecosystems and aquaculture: a colorful business with implications for human health. *Frontiers in Marine Science*.

[39] Mostafa R. E., Salama A. A. A., Abdel-Rahman R. F., Ogaly H. A. (2017). Hepato- and neuro-protective influences of biopropolis on thioacetamide-induced acute hepatic encephalopathy in rats. *Canadian Journal of Physiology and Pharmacology*.

[40] Sánchez-Valle V., Chavez-Tapia C., Uribe N. M., Méndez-Sánchez N. (2012). Role of oxidative stress and molecular changes in liver fibrosis: a review. *Current Medicinal Chemistry*.

[41] Afifi N. A., Ramadan A., El-Eraky W., Salama A. A. A., El-Fadaly A. A., Hassan A. (2016). Quercetin protects against thioacetamide induced hepatotoxicity in rats through decreased oxidative stress biomarkers, the inflammatory cytokines; (TNF-*α*), (NF-*κ* B) and DNA fragmentation. *Der Pharma Chemica*.

[42] Ma H., Chen S., Xiong H. (2020). Astaxanthin from *Haematococcus pluvialis* ameliorates the chemotherapeutic drug (doxorubicin) induced liver injury through the Keap1/Nrf2/HO-1 pathway in mice. *Food & Function*.

[43] El-Baz F. K., Salama A., Salama R. A. (2020). *Dunaliella salina* attenuates diabetic neuropathy induced by STZ in rats: involvement of thioredoxin. *BioMed Research international*.

[44] El-Baz F. K., Salama A. A. A., Hussein R. A. (2020). *Dunaliella salina* microalgae oppose thioacetamide-induced hepatic fibrosis in rats. *Toxicology Reports*.

[45] Haegele A. D., Gillette C., O’Neill C. (2000). Plasma xanthophyll carotenoids correlate inversely with indices of oxidative DNA damage and lipid peroxidation. *Cancer Epidemiology and Prevention Biomarkers*.

[46] Katsuura S., Imamura T., Bando N., Yamanishi R. (2009). *β*-Carotene and *β*-cryptoxanthin but not lutein evoke redox and immune changes in RAW264 murine macrophages. *Molecular Nutrition & Food Research*.

[47] Ni Y., Nagashimada M., Zhan L. (2015). Prevention and reversal of lipotoxicity-induced hepatic insulin resistance and steatohepatitis in mice by an antioxidant carotenoid, *β*-cryptoxanthin. *Endocrinology*.

[48] Qiu X., Gao D.-H., Xiang X. (2015). Ameliorative effects of lutein on non-alcoholic fatty liver disease in rats. *World journal of gastroenterology: WJG*.

[49] Iredale J. P. (2007). Models of liver fibrosis: exploring the dynamic nature of inflammation and repair in a solid organ. *The Journal of Clinical Investigation*.

[50] Hernández-Gea V., Ghiassi-Nejad Z., Rozenfeld R. (2012). Autophagy releases lipid that promotes fibrogenesis by activated hepatic stellate cells in mice and in human tissues. *Gastroenterology*.

[51] Friedman S. L. (2008). Mechanisms of hepatic fibrogenesis. *Gastroenterology*.

[52] Shen M., Lu J., Cheng P. (2014). Ethyl pyruvate pretreatment attenuates concanavalin a-induced autoimmune hepatitis in mice. *PLoS One*.

[53] Suzuki Y., Ohgami K., Shiratori K. (2006). Suppressive effects of astaxanthin against rat endotoxin-induced uveitis by inhibiting the NF-*κ*B signaling pathway. *Experimental Eye Research*.

[54] Fallowfield J. A. (2011). Therapeutic targets in liver fibrosis. *American Journal of Physiology-Gastrointestinal and Liver Physiology*.

[55] El-Baz F. K., Salama A., Salama R. A. A. (2019). Therapeutic effect of *Dunaliella salina* microalgae on thioacetamide- (TAA-) induced hepatic liver fibrosis in rats: role of TGF-*β*and MMP9. *BioMed research international*.

[56] Limmer A., Ohl J., Wingender G. (2005). Cross-presentation of oral antigens by liver sinusoidal endothelial cells leads to CD8 T cell tolerance. *European Journal of Immunology*.

[57] Racanelli V., Rehermann B. (2006). The liver as an immunological organ. *Hepatology*.

